The article "Green tea extract therapy diminishes hepatic fibrosis mediated by dual exposure to carbon tetrachloride and ethanol: A histopathological study" was published in 2014. Journal: Exp Ther Med.

# Green tea extract therapy diminishes hepatic fibrosis mediated by dual exposure to carbon tetrachloride and ethanol: A histopathological study

**DOI:** 10.3892/etm.2014.2158

**Published:** 2014-12-24

**Authors:** ABDEL-MAJEED SAFER, MOHAMAD AFZAL, NOMNY HANAFY, SHAKER MOUSA

**Affiliations:** 1 Department of Biological Sciences, Faculty of Science, Kuwait University, Kuwait City 13060, Kuwait; 2 The Pharmaceutical Research Institute at Albany College of Pharmacy and Health Sciences, Albany, NY 12208, USA; 3 College of Medicine, King Saud University, Riyadh 12372, Saudi Arabia

**Keywords:** green tea extract, alanine aminotransferase, aspartate aminotransferase, extracellular matrix, carbon tetrachloride plus ethanol, dual exposure, scanning electron microscopy, Masson’s trichrome stain

## Abstract

The aim of the present study was to investigate the hepatoprotective effect of green tea extract (GTE) against the hepatic fibrosis induced by carbon tetrachloride (CCl_4_), ethanol, and dual exposure to CCl_4_ plus ethanol in rats. In particular, an investigation of the three-dimensional architecture was conducted using scanning electron microscopy. Various techniques revealed that hepatic fibrosis with intermingled fibers was located between cells in the CCl_4_, ethanol and combined CCl_4_ plus ethanol groups. The hepatic fibrosis differed among the ethanol, CCl_4_ and CCl_4_ plus ethanol groups in terms of the type, thickness and distribution of fibers. The fibrotic lesions virtually disappeared in all the groups after 25 days of treatment with GTE, returning the architecture of the liver tissue to its normal status. The rats were also found to regain normal body weight and fur color, which had earlier been discolored due to weight loss. The autopsy results also showed that the animal livers returned to the normal shape and color. GTE demonstrated the same clear action in attenuating the hepatofibrosis for all three inducing treatments, by impairing collagen fibers, eliminating lipid peroxidation and returning the liver architecture to normal. GTE presents a safe therapeutic strategy for hepatic fibrosis.

## Introduction

Hepatic fibrosis is a condition in which scar formation occurs in the liver. The process occurs normally during the formation of the excessive accumulation of collagenous extracellular matrix (ECM) (1,2), or during scar tissue formation to replace normal tissue that has been lost through injury, infection or chronic liver insults (1,3–7). Specifically, hepatic fibrosis is the result of derangements in the synthesis and degradation of the matrix due to insults occurring in the mesenchymal cells that synthesize various components of the ECM, including collagen types I-VII (4,8). During our previous study on the effect of green tea extract (GTE) on the liver, kidney and stomach, the beneficial role of GTE in controlling the deleterious effects of reserpine was observed just 30 days after its administration (9). This encouraged us to study the effectiveness of GTE in ameliorating the hepatic fibrosis induced by two hepatic carcinogens, carbon tetrachloride (CCl_4_) and ethanol. Hepatic fibrosis brings about a histological change due to inflammation that causes hepatic stellate cells (HSCs) to be overactive. This activity triggers ECM synthesis and the deposition of collagen fibers in the extracellular spaces of the liver cells. In this process, blood infusion is lost and the tissue hardens, leading to liver fibrosis (10,11).

Currently, there is no effective treatment for hepatic fibrosis, and a number of patients develop a progressive form of hepatic cirrhosis. In a preliminary study, a rat model with GTE was used to control the hepatic fibrosis induced after four weeks of CCl_4_ administration (12). The rate of destruction of collagen fibers was increased. Ethanol has also been used as a hepatotoxin with a significant effect on the liver in causing hepatic fibrosis (13–15). The present study attempted to further expand on the therapeutic effects of GTE on hepatic fibrosis in rats using a model in which rats were exposed to CCl_4_ and ethanol together. The therapeutic effects of GTE on hepatic fibrosis, induced in rat liver through dual exposure to CCl_4_ plus ethanol, were investigated histologically and with three-dimensional (3D) observation using scanning electron microscopy.

## Materials and methods

### Preparation of GTE

Dried tea leaves (100 g) were powdered in a Waring blender (Waring Laboratory Supplies, Torrington, CT, USA), and extracted with double distilled water (1 l), at 85°C for 1 h. The extract was filtered through a nylon filter, and the filtrate was centrifuged at 3,000 × g for 15 min. The clear supernatant was removed and the residual pellet was agitated with distilled water, warmed at 35°C and centrifuged again. The supernatant was pooled, lyophilized and the resulting material was stored at −20°C in a screw-capped bottle.

### Schedule and groups of animals under investigation

Male albino rats (n=70), weighing 200–250 g, were obtained from the Animal Center in the Faculty of Science at Kuwait University (Kuwait City, Kuwait). The rats were maintained in an environmentally controlled room (temperature, 23±2°C; humidity, 55±10%) with a 12-h light/dark cycle and access to food and water *ad libitum.* Rats were weighed weekly using a digital balance; all the readings were recorded for statistical analysis and were used as an indication of chemical toxicity. The animals were sacrificed at the end of the treatment duration, following anesthetization with an intraperitoneal injection of 50 mg/kg pentobarbital.

### Experimental design

An experimental model of hepatic fibrosis was established chemically using ethanol and CCl_4_ separately and simultaneously. The rats were divided into seven groups as follows. GI rats (normal control) were administered a subcutaneous injection of 1 ml/100 g olive oil three times a week for three weeks. In GII and GIII, hepatic fibrosis was established using ethanol and CCl_4_. Since ethanol increases the activation of cytochrome *c*, which accentuates the metabolic activation of CCl_4_, the rats were orally administered 1 ml/100 g ethanol (25%) twice a week for one week, and subsequently 1 ml/100 g CCl_4_ (40%) by subcutaneous injection three times a week with an oral dose of 1 ml/100 g ethanol (25%) twice a week (on different days) for three weeks. The rats in GIII were subsequently treated with 1 ml/100 g GTE orally for three weeks. A hepatic fibrosis model was established in GIV and GV using ethanol alone. The rats were administered an oral dose of 1 ml/100 g ethanol (25%) twice a week for four weeks in GIV and three weeks in GV. GV rats were then administered 1 ml/100 g GTE for four weeks. In GVI and GVII, CCl_4_ was used to establish a model of hepatic fibrosis. The rats were administered a subcutaneous injection of 1 ml/100 g CCl_4_ (40%) three times a week for three weeks. GVII rats also received 1 ml/100 g GTE orally for three weeks.

### Blood sampling

Blood samples were collected by cardiac puncture following dissection. The blood was collected into dry, clean centrifuge tubes. All samples were centrifuged at 3,000 rpm for 15 min to separate the serum for the determination of aspartate aminotransferase (AST) and alanine aminotransferase (ALT).

### Histology

Liver tissues were fixed by immersion in 10% buffered neutral formalin for 18 h, processed by dehydration in an ascending series of alcohol (50, 70 and 100%) and cleared with xylene and paraffin wax. The samples were subsequently embedded in paraffin, cut into 5–7 μm sections using a rotary microtome and stained with hematoxylin and eosin (H&E).

### Tissue preparation for semi-thin sections

Liver samples from the groups of rats were fixed in 2.5% glutaraldehyde/sodium cacodylate fixative, pH 7.2 at 0–4°C for two hours, then changed to a fresh fixative and left overnight. The tissues were then transferred to sodium cacodylate/sucrose buffer, three times for 20 mins each, then to 1% OsO_4_/PO_4_ buffer for 2 h and were then blocked in Epon. Semi-thin sections (1 μm) were cut using a Leica ultra-microtome and stained with toluidine blue for observation by light microscopy and photography.

### Masson’s trichrome stain

Liver sections (7 μm) fixed in 10% buffered neutral formalin were processed for collagen fiber staining using Masson’s trichrome stain.

### 3D architecture

Sample blocks from all the groups were prepared and processed for scanning electron microscopy for a 3D-architectural observation. The blocks (~7.0 mm^3^) were fixed in 3% glutaraldehyde/cacodylate buffer (pH 7.2) using a tissue processor, then dehydrated in ethanol and freeze-dried in CO_2_. Each tissue block was then split into two, and each half of the block was fixed on a stub with the newly exposed surface facing upwards. The stubs were coated with platinum/gold using a spotter coater. A Jeol JCM 5700 Carryscope mobile scanning electron microscope (SEM; Jeol USA, Inc., Peabody, MA, USA), with a resolution of 5.0 nm, was used for attaining the SEM images.

### Biochemical analysis

AST and ALT values in all seven groups of rats were measured in serum samples using kits from Randox Laboratories Ltd. (Crumlin, Northern Ireland). The results are expressed in U/l.

### Statistical analysis

Statistical analysis was performed by one-way analysis of variance at the same time interval of weighing (P<0.05), followed by comparisons between time intervals using the least significant difference test (P<0.05), and comparing the mean ± standard deviation from each experimental group with that of the respective control group. The Pearson correlation coefficient (r) test between weight (g) and period of study (weeks) was performed. P<0.05 was considered to indicate a statistically significant difference.

## Results

### AST and ALT levels

Rats treated with GTE showed results similar to those of the control groups with normal AST and ALT levels (Fig. 1; Table I). Serum AST and ALT levels were significantly elevated in rats treated with CCl_4_ (GVI), ethanol (GIV), and CCl_4_ plus ethanol only (GII), indicating severe hepatic damage. The CCl_4_ plus GTE (GVII), ethanol plus GTE (GV), and CCl_4_ plus ethanol plus GTE (GIII) groups showed significant reductions in the levels of these two enzymes compared with those in their respective model control groups.

### Hepatic fibrosis

Hepatic fibrosis was evaluated by several criteria, including the external features, weight and gross anatomy of the rats. In the control rats, the fur color was bright white with a healthy-looking tail. For the CCl_4_-treated animals (GVI), the mean weight of the animals at the end of week 3 was 247.5±46.4 g, while following GTE administration (GVII) the mean weight reached 302.7±37.8 g (P<0.05; Table II). The weights of the animals at the end of week 4 for ethanol treatment (GIV) were 320.4±42.0 g, while following GTE administration (GV) they reached 271.6±55.0 g (P<0.05; Table III). However, at the end of week 4, the mean weight of the animals in the ethanol plus CCl_4_-treated group (GII) was 251.2±58.1 g, while following GTE administration (GIII) they reached 271.6±55.0 g (P<0.05; Table IV). Furthermore, to evaluate whether normal growth was observed within the study period, a two-tailed Pearson correlation coefficient test was used and the results are shown in Table V. There was significant increase in weight within the study period (normal growth; r=0.68, P<0.001) in the control group, but the increase in weight in the CCl_4_ group was not significant within the period of study, indicating that CCl_4_ suppresses growth. Gross anatomy at the onset of postmortem and prior to organ excision showed the liver of a rat from GI to exhibit a normal brownish-red color with minimal loci of fat (Fig. 2A). In the H&E-stained paraffin and toluidine blue-stained Epon sections, the control group showed normal tissue and cell architecture (Fig. 2B and C). This was also observed in the sections with Masson’s trichrome staining, which is specifically for collagen fibers (Fig. 2D).

In the CCl_4_ plus ethanol group (GII) the external features of the rat showed fur with yellowish to brown coloration with an abnormally dark-colored tail. At the onset of postmortem and prior to organ excision, the liver appeared fibrotic and orange in color and was topped with thick fat (Fig. 3A). The H&E-stained paraffin and toluidine blue-stained Epon sections exhibited pathological features, notably including the formation of an extensive amount of extracellular fibrous materials in the parenchyma of the liver (Fig. 3B and C). Fibrous materials (collagen fibers) were clearly observed in the Masson’s trichrome-stained sections as shades of blue-green-stained structures (Fig. 3D). Profuse collagen fiber deposits filled a number of areas in the extracellular spaces of the liver parenchyma of GII rats. The fibers varied in thickness from 250 to 1,000 nm (Fig. 4). Other pathological features observed were the destruction of the lobular architecture, inflammation, foamy vacuolated cytoplasm, necrosis, fatty cells, steatosis, nuclear shrinkage, abnormal tri- and tetra-polar divisions, nuclear karyorrhesis, nuclear karyolysis, nuclear hyperchromatism, dead cells, thickening of the portal vein and triad, hypertension of arterioles, nuclear hyperchromatism, nuclear fragmentation, condensed eosinophilic protein, hyperactive Kupffer cells and proliferation of HSCs (data not shown). The Carryscope SEM facilitated the observation of two types of fibrous materials in the ECM: Thick fibers (average 312.41 nm) always appeared in the CCl_4_-treated liver (GII) and thin, fluffy fibers (average 169.71 nm) always appeared in the ethanol-treated liver (GIV; Fig. 4).

### Effects of GTE treatment

Rats in the CCl_4_ plus ethanol plus GTE group (GIII) exhibited almost complete restoration of liver function. Externally, the normal, healthy, bright color of the rat, including the tail, was restored. In the gross morphology, the liver looked fairly normal, exhibiting a bright red color and the absence of fat (Fig. 5A). Fibrous materials and lipid droplets were not present as demonstrated in the H&E-stained paraffin or toluidine blue-stained Epon sections (Fig. 5B and C). Masson’s trichrome-stained sections of liver tissue exhibited prominent restoration of liver morphology. The fibrous materials completely disappeared from the ECM and there were no signs of lipid droplets (Fig. 5D). A 3-D architectural observation was performed with the Carryscope SEM of the fractured surfaces of the CCl_4_ plus ethanol-treated (GII) liver tissue. The images showed morphologically two types of collagen fiber strands: Thick and dark, and thin yet puffy (Fig. 6A). However, in the CCl_4_ plus ethanol plus GTE-treated group (GIII) the image was completely devoid of fibers (Fig. 6B). In the CCl_4_-treated group (GVI) collagen fibers type were present due to CCl_4_ (Fig. 6C, white arrows). In the CCl_4_ plus GTE-treated group (GVII) the collagen fibers disappeared (Fig. 6D). In the ethanol-treated group (GIV) collagen fibers type formed due to the ethanol that was present (Fig. 6E). In the ethanol plus GTE-treated group (GV) no collagen fibers type formed (Fig. 6F).

## Discussion

Hepatic fibrosis is a global challenge. In our previous study, it was observed that GTE attenuated the hepatic fibrosis mediated by CCl_4_ in rats (12). In the present study, liver fibrosis was induced in a group of rats with a dual exposure to CCl_4_ plus ethanol. Administration of alcohol with repetitive CCl_4_ ingestion enhances the toxicity of CCl_4_ in rats (16). Other groups of rats were also treated with CCl_4_ alone and ethanol alone as described in Materials and methods. After 25 days, immediately prior to dissection, the animals appeared fragile and thin with pale yellow hairs, particularly those with the dual exposure. This was in contrast to the control animals and those that subsequently received GTE treatment. During autopsy, the CCl_4_ plus ethanol-treated liver showed a typical fibrotic orange color instead of the normal reddish-brown color. Fat deposition and color intensity were increased compared with those in the animals that were treated with CCl_4_ or ethanol alone. The weights of the animals steeply declined with the onset of the CCl_4_ treatments, and gradually increased with GTE administration between the first and third weeks. Towards the end of the assigned experiment on week four, almost all the GTE-treated animals returned to the normal body weight, similar to that of the control group (P<0.05). By contrast, the weights of the animals increased with the onset of ethanol and gradually decreased with GTE to become in line with those of the control group (P<0.05). The CCl_4_ group treated with GTE showed normal growth (r=0.5, P=0.009). In the group treated with ethanol, the weight of the rats increased rapidly within the period of the study (r=0.41, P=0.01) and an increase in weight was also observed in the ethanol plus GTE group (r=0.18, P=0.27). Rats treated with ethanol plus CCl_4_ showed a reduction in weight with time as the result of the effect of the CCl_4_, but this effect was slightly reversed by the ethanol and therefore gave a non-significant reduction in weight (r=−0.20, P=0.25). The effect of GTE on the ethanol plus CCl_4_ group showed a shift in weight toward the normal weight (r=−0.02, P=0.92).

Histological observations of liver tissues using H&E and toluidine blue staining of sections all coincided with the external status of the animals and the aforementioned autopsy features. Histopathological changes were clear in the H&E and toluidine blue liver sections including the destruction of lobular architecture, inflammation, large foamy vacuolated cytoplasm, necrosis, large fatty cells, steatosis, nuclear shrinkage, abnormal tri- and tetra-polar divisions, nuclear karyorrhesis, nuclear karyolysis, nuclear hyperchromatism, dead cells, thickening of the portal vein and triad, hypertension of arterioles, nuclear hyperchromatism, nuclear fragmentation, condensed eosinophilic protein, hyperactive Kupffer cells and proliferation of HSCs (11). However, the majority of these pathological features were markedly reduced following GTE administration. Notably, the cytoplasmic vacuolation and large fatty cells disappeared, a finding that was not only observed in the gross morphology but also in the H&E- and toluidine blue-stained sections. It has been shown in studies using mice that dietary GTE and regular exercise, if combined, stimulate fat catabolism not only in the liver but also in skeletal muscle, and attenuate high-fat diet-induced obesity more effectively than each alone (10), as well as altering plasma lipids, glucose and liver lipids (17). The Masson’s trichrome-stained liver tissues clearly showed the intermingled fibrous materials in the CCl_4_ plus ethanol-treated liver as blue-green fibrous structures among the cells and surrounding the blood vessels. These fibers were not present in the GTE-treated groups, which appeared similar to the control group. The surface topography of the fractured surface of the liver blocks when observed under the SEM also showed how the types of fibers of varied thickness and direction intermingled in the liver parenchyma around the hepatocytes (13).

A number of studies have shown that during hepatic fibrosis, proteins including collagen types I and III proliferate (9). Administration of GTE either simultaneously or following CCl_4_, ethanol or CCl_4_ plus ethanol administration prevented hepatic fibrosis. This may indicate that GTE inhibits the proliferation of HSCs (4,15). All GTE-treated groups showed a great effect of GTE in removing almost all the fibers observed in an area when compared with the CCl_4_ plus ethanol group. Notably, two types of fibrous material have been recognized. Thick fibers (average 312.41 nm) were always shown in the CCl_4_-treated liver and thin, fluffy fibers (average 169.71 nm) always appeared in the ethanol-treated liver, in reference to the normal range of 800–2,400 nm (14), which indicated hepatic injury (4,15). These alterations were clearly reduced following treatment with GTE.

The innovation from the present study is that GTE inhibits the damaging effects caused by the oxidative stress of CCl_4_, ethanol, or even combined CCl_4_ plus ethanol on the liver cells, and the ECM components are comparable to those of the liver and kidney cells of previous studies in which reserpine was used (7,9). Thus GTE significantly reduced cellular leakage of hepatocyte ALT and AST and apparently improved cell viability. Severe hepatic lesions induced by the dual action of CCl_4_ plus ethanol were markedly improved by the administration of GTE. GTE also reduces inflammation and destruction of the liver architecture and the downregulation of the platelet-derived growth factor-β receptor (6); therefore, it prevents the development of CCl_4_ plus ethanol-induced hepatic fibrosis in rats. This suggests that the polyhydroxy phenols (catechins) of green tea exhibit strong antioxidant activity against reactive oxygen species, and have beneficial health effects by repairing the structure and function of the ECM to a significant degree, presumably through (-)-epigallocatechin gallate, the active ingredient in green tea that inhibits the activation of receptor tyrosine kinases associated with HSCs (11). Green tea may lead to improved health by reducing oxidative stress; however, this varies according to toxin and organs (4,9,18–26). The present study demonstrates that GTE exhibits anti-fibrotic and anti-oxidative effects in rats in which fibrosis is induced by dual exposure to CCl_4_ plus ethanol, and thus may be used as a therapeutic option and defensive measure in the prevention of hepatic fibrosis.

## Figures and Tables

**Figure 1:** AST and ALT levels. (A) AST levels and (B) ALT levels in rats treated with CCl_4_, ethanol, and CCl_4_ plus ethanol in the presence and absence of GTE. Groups: GI, normal control; GII, CCl_4_ plus ethanol; GIII, CCl_4_ plus ethanol plus GTE; GIV, ethanol; GV, ethanol plus GTE; GVI, CCl_4_; GVII, CCl_4_ plus GTE. AST, aspartate aminotransferase; ALT, alanine aminotransferase; SD, standard deviation; CCl_4_, carbon tetrachloride; GTE, green tea extract.

**Figure 2:** Images of the liver of a rat from GI. (A) Gross morphology of the healthy liver of the rat with a normal reddish-brown color. (B) Hematoxylin and eosin- (magnification, ×240), (C) toluidine blue- (magnification, ×300) and (D) Masson’s trichrome- (magnification, ×400) stained sections of the liver. GI, normal control group.

**Figure 3:** Images from a GII rat. (A) Abnormal fatty liver of a GII rat. (B) Hematoxylin and eosin-stained section of the liver. Intermingled fibrous materials are observed among the hepatocytes (large arrows) as well as vacuolations and lipid droplets (small arrows; magnification, ×100). (C) Toluidine blue-stained section of the liver. Intermingled fibrous materials are observed among the hepatocytes (large arrows) as well as vacuolations and lipid droplets (small arrows; magnification, ×1,000). (D) Masson’s trichrome-stained section of the liver showing the accumulation of collagen fibers in the extracellular matrix (white arrows); the image shows a number of areas of lipid droplets and inflammation (magnification, ×400). GII, carbon tetrachloride plus ethanol group.

**Figure 4:** Thickness of collagen fibers due to the effects of ethanol and CCl_4_. Scanning electron microscope images showing the thickness (nm) of collagen fibers formed in the extracellular matrix of the rat liver due to (A) CCl_4_ administration and (B) ethanol administration. CCl_4_, carbon tetrachloride.

**Figure 5:** Images of a GIII rat. (A) Gross morphology of the liver of a GIII rat with a normal reddish-brown color. (B) Hematoxylin and eosin-stained section of the liver. The image is devoid of fibers and lipid droplets (magnification, ×200). (C) Toluidine blue-stained section of the liver. The image is devoid of fibers and lipid droplets (magnification, ×1,000). (D) Masson’s trichrome-stained section of the liver with no collagen fibers in the extracellular matrix. The image also lacks lipid droplets (magnification, ×400). GIII, carbon tetrachloride plus ethanol plus green tea extract group.

**Figure 6:** Scanning electron microscope images of the rat liver extracellular matrix. (A) GII rat with collagen fiber formation due to CCl_4_ (white arrows) and ethanol (black arrows). (B) GIII rat with reduced presence of collagen fibers. (C) GVI rat with collagen fiber formation due to CCl_4_ (white arrows). (D) GVII rat with reduced presence of collagen fibers. (E) GIV rat with collagen fiber formation (white arrows). (F) GV rat with no collagen fibers. Groups: GII, CCl_4_ plus ethanol; GIII, CCl_4_ plus ethanol plus GTE; GIV, ethanol; GV, ethanol plus GTE; GVI, CCl_4_; GVII, CCl_4_ plus GTE. CCl_4_, carbon tetrachloride; GTE, green tea extract.

**Table I:** ALT and AST activity levels in the studied groups.

Activity levels (U/I)	GI	GII	GIII	GIV	GV	GVI	GVII
ALT	22.0±2.6	27.5±2.0^b^	22.0±2.2^a^	26.5±1.9^b^	20.3±1.6^a^	38.5±2.5^b^	22.0±2.1^a^
AST	31.4±4.9	41.6±7.5^b^	30.3±2.9^a^	40.0±4.9^b^	28.6±2.0^a^	57.5±4.4^b^	40.0±4.9^a^

a P<0.05 vs. the respective model control without GTE treatment;

b P<0.05 vs. the normal control (using the least significant difference test). Data are presented as the mean ± standard deviation.

Groups: GI, normal control; GII, CCl_4_ plus ethanol; GIII, CCl_4_ plus ethanol plus GTE; GIV, ethanol; GV, ethanol plus GTE; GVI, CCl_4_; GVII, CCl_4_ plus GTE. ALT, alanine aminotransferase; AST, aspartate aminotransferase; CCl_4_, carbon tetrachloride; GTE, green tea extract.

**Table II:** Rat weights in the control, CCl_4_ and CCl_4_ plus GTE groups over three weeks.

Week	Control group	CCl_4_ group	CCl_4_ plus GTE group	P-value^a^
1	213.0±22.8	246.0±38.4	246.6±45.0	0.0816
2	248.1±26.3	256.5±41.4	273.2±43.4	0.3355
3	262.5±26.2	247.5±46.4	302.7±37.8^b^	0.0086

a The P-value was determined by one-way analysis of variance and considered significant if P<0.05;

b P<0.05 versus the control group (using the least significant difference test). N=10 in each group. Data are presented as the mean ± standard deviation.

GTE, green tea extract; CCl_4_, carbon tetrachloride.

**Table III:** Rat weights in the control, ethanol and ethanol plus GTE groups over four weeks.

Week	Control group	Ethanol group	Ethanol plus GTE group	P-value^a^
1	213.0±22.8	276.6±28.9^b^	246.9±25.8^b^	<0.0001
2	248.1±26.3	300.4±37.4^b^	277.9±41.3	0.0105
3	262.5±26.2	311.4±39.4^c^	272.5±47.8	0.0220
4	281.9±33.3	320.4±42.0^c^	271.6±55.0	0.0499

a The P-value was determined by one-way analysis of variance and considered significant if P<0.05;

b P<0.05 versus the control group;

c significant versus the ethanol plus GTE group (using the least significant difference test). N=10 in each group. Data are presented as the mean ± standard deviation.

GTE, green tea extract.

**Table IV:** Rat weights in the control, CCl_4_ plus ethanol and CCl_4_ plus ethanol plus GTE groups over four weeks.

Week	Control group	CCl_4_ plus ethanol group	CCl_4_ plus ethanol plus GTE group	P-value^a^
1	213.0±22.8	275.6±45.1^b^	271.8±36.4^b^	0.0007
2	248.1±26.3	274.7±46.2	277.9±41.3	0.1900
3	262.5±26.2	256.2±57.3	272.5±47.5	0.7459
4	281.9±33.3	251.2±58.1	271.6±55.0	0.4563

a The P-value was determined by one-way analysis of variance and considered significant if P<0.05;

b significant versus the control group (using the least significant difference test). N=10 in each group with the exception of weeks 3 and 4 of the CCl_4_ plus ethanol group (n=7, 3 rats died). Data are presented as the mean ± standard deviation.

GTE, green tea extract; CCl_4_, carbon tetrachloride.

**Table V:** Two-tailed Pearson correlation coefficient test between rat weight (g) and period of study (weeks).

Group	r	P-value
Control (n=40)	0.68	<0.001
CCl_4_ (n=30)	0.02	0.94
CCl_4_ plus GTE (n=30)	0.50	0.009
Ethanol (n=40)	0.41	0.01
Ethanol plus GTE (n=40)	0.18	0.27
CCl_4_ plus ethanol (n=34)	−0.20	0.25
CCl_4_ plus ethanol plus GTE (n=40)	−0.02	0.92

r, Pearson correlation coefficient; CCl_4_, carbon tetrachloride; GTE, green tea extract.
